# Diagnosis of Hypersensitivity Induced by Antituberculosis Drugs

**DOI:** 10.1155/2021/6455659

**Published:** 2021-12-20

**Authors:** Yuqing Wu, Guangming Xiao, Peilan Zong, Guoqiang Jiang, Yongmei Liao, Zhou Liu, Yanhong Zhou

**Affiliations:** ^1^Department of Tuberculosis, Jiangxi Chest Hospital, Nanchang 330006, Jiangxi, China; ^2^Jiangxi Clinical Research Center for Infectious Diseases, Nanchang 330006, Jiangxi, China

## Abstract

**Objective:**

To explore the clinical value of the specific plasma cell detection and specific T lymphocyte detection test in diagnosing hypersensitivity caused by antituberculosis drugs.

**Methods:**

A total of 266 patients with pulmonary tuberculosis who developed hypersensitivity during the treatment of primary pulmonary tuberculosis in our hospital and 266 patients without hypersensitivity during the treatment of pulmonary tuberculosis in our hospital were selected as the control group. The admission time is from January 2013 to June 2020. The specific plasma cell test and specific T lymphocyte test were used as the criteria to determine which drugs induced hypersensitivity, and the diagnostic value of these two methods in the diagnosis of hypersensitivity induced by four first-line antituberculosis drugs (isoniazid (INH), ethambutol (EMB), rifampicin (RFP), and pyrazinamide (PZA)) was analyzed.

**Results:**

The sensitivity of the specific plasma cell test in the diagnosis of hypersensitivity induced by INH, EMB, RFP, and PZA was 63.42%, 51.20%, 47.81%, and 56.37%, respectively, and the specificity was 95.33%, 99.87%, 96.52%, and 99.99%, respectively. The sensitivity of the specific T lymphocyte test in the diagnosis of hypersensitivity induced by INH, EMB, RFP, and PZA was 66.47%, 52.88%, 49.91%, and 58.54%, respectively, and the specificity was 97.28%, 99.99%, 98.38%, and 100.00%, respectively.

**Conclusion:**

The specific plasma cell test and specific T lymphocyte test have high specificity in the diagnosis of hypersensitivity caused by antituberculosis drugs, and the specific T lymphocyte test is better than the specific plasma cell test. It is of great significance to guide the clinical application of antituberculosis drugs.

## 1. Introduction

Tuberculosis is one of the infectious diseases that threaten human health [1]. According to WHO statistics, there were 10.4 million new tuberculosis cases worldwide before 2016, with about 1.6 million deaths [2]. China is still one of the 30 countries with high TB burden in the world [3], with about 900000 new TB patients every year, ranking third in the world [4]. At present, the standard treatment regimen consisting of isoniazid (INH), rifampicin (RFP), ethambutol (EMB), and pyrazinamide (PZA) can effectively treat most newly diagnosed tuberculosis patients [5, 6]. However, these antituberculosis chemical drugs may cause a variety of adverse reactions. Hypersensitivity is one of the common adverse reactions, which is often called drug allergy in clinics [7–9]. Drug hypersensitivity syndrome (DIHS) is a severe allergic reaction, which is characterized by fever, rash, enlarged lymph nodes, eosinophilia, proliferation of atypical lymphocytes in peripheral blood, impaired liver function, or other organ function damage. Its incidence is 1 : 10000–1:1000, and the case fatality rate is as high as 10% [10, 11]. Studies have shown that DIHS caused by antituberculosis drug (ATD) accounts for 13.3% of all DIHS, ranking third [12]. ATD-induced DIHS has its own characteristics; it is a combination of drugs; it is difficult to determine sensitizing drugs, once the first-line ATD is sensitized; it is difficult to choose alternative treatment, resulting in tuberculosis drug resistance and treatment failure. At present, the commonly used method for the diagnosis of hypersensitivity caused by antituberculosis drugs is the drug lymphocyte stimulation test, which has a high specificity in the diagnosis of patients with hypersensitivity caused by antituberculosis drugs, although the sensitivity is slightly low. However, it is still of great significance to guide the clinical use of drugs.

According to the Gell–Coombs classification method, allergic reactions are divided into fast hairstyle (I type), cytotoxic (II type), immune complex (IV type), delayed-type hypersensitivity (III type), and allergic reactions caused by antituberculosis drugs mainly for delayed-type hypersensitivity (V type) [13]. Current clinical diagnosis of allergic reactions caused by antituberculosis drugs mainly rely on the drug test (DPT), due to anti-tb drugs are often combined application; however, it can cause allergic reactions or even again exfoliative dermatitis; prolonged hospitalization in the patients not only increase the pain of the patients at the same time but also to a certain extent a blow to treat disease of confidence, hardly conducive to the prevention and control of tuberculosis in China [14]. China has the second largest TB burden in the world [15], How to quickly, safely, and accurately identify drugs that cause hypersensitivity reactions is a problem that clinicians urgently need to solve. The purpose of this study is to explore the sensitivity and specificity of the specific plasma cell test and specific T lymphocyte test in the diagnosis of antituberculosis drug-induced hypersensitivity, so as to lay a foundation for the comprehensive in vitro detection of antituberculosis drug-induced hypersensitivity in the future.

## 2. Materials and Methods

### 2.1. Study Design and Participants

#### 2.1.1. General Information

A total of 266 patients who developed hypersensitivity during the treatment of pulmonary tuberculosis in our hospital from January 2013 to June 2020 were selected (group A). 266 patients without hypersensitivity during the treatment of pulmonary tuberculosis in our hospital were selected as the control group (group B). There were 266 patients in group A, aged from 22 to 67 years old, with an average age of (41.5 ± 5.3) years. 266 patients in group B served as the control group, aged from 18 to 69 years old, with an average age of (40.9 ± 6.4) years. There was no significant difference in sex (*χ*^2^ = 0.823) and age (*t* = 1.962) between the two groups (*P* > 0.05). This study was examined and approved by the ethics committee of our hospital, and all the patients had informed consent.

#### 2.1.2. Inclusion Criteria

(1) It conforms to the relevant diagnostic criteria of newly treated pulmonary tuberculosis in the tuberculosis diagnosis and treatment guidelines of Tuberculosis Branch of Chinese Medical Association; and (2) the clinical manifestation and laboratory examination accorded with the diagnosis of drug-induced hypersensitivity in Clinical Dermatology, which was jointly diagnosed by two specialists.

#### 2.1.3. Exclusion Criteria

(1) Complicated with HIV infection; (2) complicated with chronic kidney disease, diabetes, hematopoietic system diseases, and autoimmune-related diseases; (3) taking antituberculosis treatment while taking other disease treatment drugs; (4) misdiagnosis and misacceptance; and (5) immunosuppressant was used in the process of antiallergic treatment.

## 3. Methods

### 3.1. Preparation of Experimental Drugs

The single dose of antituberculosis drugs (INH, EMB, RFP, and PZA) taken by the patient was dissolved in 5 ml double distilled water or dimethyl sulfoxide (DMSO) by severe concussion; then, the bacteria were removed by 0.22 *μ*m filter and diluted into three concentration gradients (1 : 10, 1 : 100, and 1 : 1000) in the RPMI-1640 culture medium.

### 3.2. Isolation of PBMC from Peripheral Blood Mononuclear Cells

After the patient was enrolled in the group, 10 ml venous blood was collected for preparation PBMC, 1×phosphate buffer (PBS) was isolated from heparin anticoagulant blood samples by density gradient centrifugation, resuspended in 2 ml RPMI-1640 culture medium (containing 10% fetal bovine serum + penicillin streptomycin) and counted, and the cell concentration was adjusted to 1×10 ^6^/ml. 1 × 10^5^/100 *μ*l PBMC was added to each well of 96-well plate, and then, 5 *μ*l of preprepared stimulant drug was added. Negative control holes (drug dissolving medium + culture medium + PBMC), positive control holes (phytohemagglutinin (PHA) 5 *μ*g/ml + culture medium + PBMC), and zeroing holes (only culture medium) were set up, and there were 3 compound holes in each group. At the same time, the anticoagulant blood samples of 1 patient in the control group were randomly selected for the same experiment. The culture plate was placed at 37°C and cultured in 5% CO_2_ incubator for 60 h, and the cell growth was observed under the inverted microscope.

### 3.3. Specific Plasma Cell Detection and Specific T Lymphocyte Detection

Flow cytometry (BD company FACSCaliburTM) was used to detect specific plasma cells and specific T lymphocytes. According to the requirements of the reagent instructions, 20 *μ*L of TriTESTCD4/CD8/CD3 reagent and 50 *μ*L of peripheral anticoagulant were added into the counter tube to mix evenly. After incubating 15 min without light, 450 ml of hemolytic agent was added, mixed, and incubated without light for 15 min and then detected on the computer.

### 3.4. Determination of Drugs Leading to Hypersensitivity

After the symptoms of hypersensitivity were relieved after drug withdrawal and the results of specific plasma cell test and specific T lymphocyte test were determined, DPT (the gold standard for clinical judgment of which drug caused hypersensitivity) was performed. The interval between each drug was 3-4 d. Once DPT was positive during the test period, it could be determined as the hypersensitivity of the drug.

### 3.5. Statistical Method

SPSS25.0 statistical software was used for data analysis. The measurement data were expressed by (‾*x* ± *s*), the two groups were compared with two independent samples *t*-test, and the counting data were compared with the *χ*^2^ test. The difference was statistically significant (*P* < 0.05).

## 4. Results

### 4.1. Diagnostic Value of Specific Plasma Cell Detection and Specific T Lymphocyte Detection Test in Antituberculosis Drug-Induced Hypersensitivity

A total of 272 cases of antituberculosis drug-induced hypersensitivity were detected by DPT (4 cases were caused by EMB, PZA, and RFP and 2 cases were induced by EMB and RFP). A total of 5 cases of hypersensitivity induced by two antituberculosis drugs were detected by the specific plasma cell test and specific T lymphocyte test (3 cases by EMB and PZA and 2 cases by INH and RFP).

The sensitivity of the specific plasma cell test in the diagnosis of hypersensitivity induced by INH, EMB, RFP, and PZA was 63.42%, 51.20%, 47.81%, and 56.37%, respectively, and the specificity was 95.33%, 99.87%, 96.52%, and 99.99%, respectively (Tables 1–4).

The sensitivity of the specific T lymphocyte test in the diagnosis of hypersensitivity induced by INH, EMB, RFP, and PZA was 66.47%, 52.88%, 49.91%, and 58.54%, respectively, and the specificity was 97.28%, 99.99%, 98.38%, and 100.00%, respectively (Tables 5–8).

## 5. Discussion

Hypersensitivity reaction is one of the most common adverse reactions of antituberculosis drugs at present, and the clinical symptoms of DIHS caused by ATD are various [16, 17], including the following typical characteristics: (1) delayed drug anaphylaxis, that is, adverse reactions occur within 2 weeks to 3 months after the use of ATD; (2) clinical manifestations and laboratory tests are similar to virus infection; and (3) symptoms persist or worsen after withdrawal of related drugs. Involvement of internal organs is a prominent feature of DIHS. Studies by Husain et al. [18] have shown that drug-induced DIHS may sometimes involve specific organs, such as penicillins, allopurinol, and antiepileptic drugs. ATD is prone to liver injury, including drug direct toxicity and immune-mediated liver injury, that is, hypersensitive liver injury, liver injury caused by lipid peroxidation [19]. In the reported DIHS caused by ATD, visceral organs are involved extensively and severely, and there is no obvious organ specificity, which can lead to liver damage, polymyositis, myocarditis, pneumonia, and acute renal failure [20, 21]. Even in hemophagocytic syndrome antibiotics are ineffective when DIHS is involved in the lungs, but lung lesions are absorbed after glucocorticoid treatment. The pathological changes of the skin are prominent; different from drug eruptions such as severe pleomorphic erythema and toxic epidermal necrolysis, urticaria and macular papules are the most common [22].

The pathogenesis may be related to virus activation, abnormal immune response, and genetic susceptibility factors. It can be explained that in susceptible individuals [23], with certain (HLA) alleles of human leukocyte antigen, taking related drugs for a certain time and dose, due to the deficiency of drug metabolic enzymes and the accumulation of toxic metabolites, lead to the formation of new antigens between semiantigens, intermediate reaction metabolites, and tissue macromolecules, and the costimulatory signal pathway is induced by antigen presenting cells; thus, the potential virus is activated and cloned T cells are expanded. T cells produce cytokines, infiltrate into the skin and other organ functions, and increase the number of eosinophils in peripheral blood and tissue [24]. Some studies have pointed out that 12H-R-Z-E regimen can significantly provide the success rate of treatment, greatly reduce the loss of follow-up rate of patients, effectively reduce hypersensitivity reactions, and help to reduce other adverse drug reactions and reduce the mortality of patients. The most effective way to deal with drug hypersensitivity is to temporarily suspend treatment and wait for the patient's hypersensitivity to recover to offspring with other therapeutic drugs with different chemical structures. This will not only prolong the length of stay of patients but also aggravate the pain of patients, undermine patients' confidence in treating the disease, and even cause patients to give up treatment, which is not conducive to the prevention and control of tuberculosis in our country. Therefore, to find a rapid, accurate, and safe detection method of antituberculosis drugs that lead to hypersensitivity is the common direction of tuberculosis clinical staff.

This study analyzed the diagnostic value of hypersensitivity caused by four first-line antituberculosis drugs (INH, EMB, RFP, and PZA) with specific plasma cell detection and specific T lymphocyte detection. The results showed that the specific plasma cell detection and specific T lymphocyte detection test has certain significance in the diagnosis of hypersensitivity caused by antituberculosis drugs. It is mainly characterized by high specificity, but the sensitivity is generally low. Consider the following possible reasons. (1) Drugs: the pathological mechanism of hypersensitivity reactions is complicated, and T lymphocyte immunity cannot fully cover the causes of hypersensitivity reactions caused by various drugs; (2) the patients in this study stay in the hospital within a short period of time after the rash occurs. Take venous blood, considering the influence of the drug washout period. In the future, a variety of in vitro detection methods will be combined in different periods after the hypersensitivity reaction occurs in patients, and the sensitivity is expected to be improved. This study found that the sensitivity and specificity of the specific T lymphocyte test are higher than that of the specific plasma cell test (the sensitivity of the specific plasma cell test to diagnose hypersensitivity caused by INH, EMB, RFP, and PZA is 63.42%, 51.20%, 47.81%, and 56.37%, respectively, with specificities of 95.33%, 99.87%, 96.52%, and 99.99%, respectively. The sensitivity of specific T lymphocyte detection tests to diagnose hypersensitivity caused by INH, EMB, RFP, and PZA are, respectively, 66.47%, 52.88%, 49.91%, and 58.54% and the specificities are, respectively, 97.28%, 99.99%, 98.38%, and 100.00%, but this article did not compare the correlation and difference, and this research experiment still needs more. This is further confirmed by a large research population.

There are many adverse reactions of ATD. For severe adverse drug reactions such as DIHS, more attention should be paid to the study of susceptible genes, specific viruses, cytokines, and new biomarkers. Attention should be paid to the adverse reactions of glucocorticoids in the course of treatment. Considering the risk of the drug stimulation test, more safe and effective laboratory examination methods are needed. To sum up, the specific plasma cell test and specific T lymphocyte test have high specificity in the diagnosis of antituberculosis drug-induced hypersensitivity; although the sensitivity is slightly lower, but it is still of great significance in guiding clinical drug use.

## Figures and Tables

**Table 1:** Diagnostic value of the specific plasma cell test in INH-induced hypersensitivity.

Specific plasma cell test	DPT		Total
	Positive	Negative	
Positive	88	15	103
Negative	40	389	431
Total	128	404	532

**Table 2:** Diagnostic value of the specific plasma cell test in EMB-induced hypersensitivity.

Specific plasma cell test	DPT		Total
	Positive	Negative	
Positive	70	28	98
Negative	84	350	434
Total	154	378	532

**Table 3:** Diagnostic value of the specific plasma cell test in RFP-induced hypersensitivity.

Specific plasma cell test	DPT		Total
	Positive	Negative	
Positive	65	30	95
Negative	95	342	437
Total	160	372	532

**Table 4:** Diagnostic value of the specific plasma cell test in PZA-induced hypersensitivity.

Specific plasma cell test	DPT		Total
	Positive	Negative	
Positive	77	20	97
Negative	73	362	435
Total	150	382	532

**Table 5:** The diagnostic value of the specific T lymphocyte test in INH-induced hypersensitivity.

Specific T lymphocyte test	DPT		Total
	Positive	Negative	
Positive	94	13	107
Negative	28	397	425
Total	122	410	532

**Table 6:** Diagnostic value of the specific T lymphocyte test in EMB-induced hypersensitivity.

Specific T lymphocyte test	DPT		Total
	Positive	Negative	
Positive	72	30	102
Negative	86	344	430
Total	158	374	532

**Table 7:** Diagnostic value of the specific T lymphocyte test in RFP-induced hypersensitivity.

Specific T lymphocyte test	DPT		Total
	Positive	Negative	
Positive	60	34	94
Negative	103	335	438
Total	163	369	532

**Table 8:** The diagnostic value of the specific T lymphocyte test in PZA-induced hypersensitivity.

Specific T lymphocyte test	DPT		Total
	Positive	Negative	
Positive	79	34	113
Negative	70	349	419
Total	149	383	532

## Data Availability

The analyzed datasets generated during the study are available from the corresponding author upon request.
